# The Effect of Osteoprotectin (OPG)/Receptor Activator of Nuclear Factor-*κ*B Ligand (RANKL)/Receptor Activator of Nuclear Factor-*κ*B (RANK) Gene Methylation on Aortic Valve Calcified

**DOI:** 10.1155/2022/1592576

**Published:** 2022-08-12

**Authors:** Wei Luo, Yanqiu Song, Jing Wang, Xia Yang, Zuocheng Li, Hongliang Cong

**Affiliations:** ^1^Department of Cardiovascular Disease, Tianjin Chest Hospital, Tianjin 300222, China; ^2^Angiocardiopathy Institute, Tianjin Chest Hospital, Tianjin 300222, China; ^3^Department of Pathology, Tianjin Chest Hospital, Tianjin 300222, China

## Abstract

To evaluate the effect of the methylation of osteoprotectin (OPG)/receptor activator of nuclear factor-*κ*B ligand (RANKL)/receptor activator of nuclear factor-*κ*B (RANK) pathway on aortic valve calcification, the aortic valve tissue was collected from 38 aortic stenosis (AS) patients who underwent valve replacement. OPG and RANKL gene methylation, RT-PCR, and ELISA were performed. Hematoxylin-eosin staining (HE), alizarin red-S staining, and immunohistochemically staining of OPG, RANKL, and CD68 were simultaneously performed. The patients were divided into noncalcified group (*n* = 21) and calcified group (*n* = 17). The methylation rate of OPG gene in noncalcified group was higher than that in calcified group (*P* = 0.027). The methylation degree of RANKL gene was generally lower, but the noncalcified group was still higher than that in the calcified group (*P* = 0.025). RT-PCR analysis showed that the mRNA expression of OPG and RANKL was higher in calcified group than in noncalcified group (*P* = 0.007 and *P* = 0.036, respectively), and the mRNA expression was negatively correlated with the gene methylation rate. The protein expression of OPG and RANKL was detected by immunohistochemistry and ELISA, showing significantly increased in calcified group (*P* = 0.004 and *P* = 0.042, respectively). Soluble RANKL (sRANKL) in CD68-positive group was significantly different from that in negative group (0.1243 ± 0.0321 vs 0.0984 ± 0.0218 pg/mL, *P* = 0.007). There was no significant difference in OPG value between positive group (1.9411 ± 0.4554 ng/mL) and negative group (1.8422 ± 0.5218 ng/mL, *P* = 0.587). In conclusion, the degree of methylation of OPG and RANKL genes may play an important role in regulating valve calcification in AS patients.

## 1. Introduction

Calcific aortic valve disease (CAVD) is a slow, progressive disorder, characterized by fibrosis, sclerosis, and calcium deposits of aortic valve and surrounding tissues [1]. By far, CAVD, as the most prevalent form of aortic stenosis (AS), is cumulatively widespread globally with significant high morbidity and mortality and has become a growing public health problem [2]. CAVD mainly shows two major kinds of functional impairments: one manifested as mild valve thickening without obstruction of blood flow and the other manifested as severe calcification with damaged leaflet motion [3, 4]. AS is the most prevalent valvular heart disease and the third most common cardiovascular condition after coronary artery disease and hypertension [2, 5]. In the past 50 years, dramatic changes have taken place in the treatment of calcified AS. However, no drug therapy has been shown to reduce the progression of calcified AS or the adverse effects on patients' prognosis. Therefore, it is very important to understand the mechanisms related to the progression of AS, which may help to explore effective ways to treat AS patients.

A number of basic science and clinical studies have clearly indicated that aortic valve calcification is an active biological process with strong genetic components, involving mechanisms similar to osteogenesis [6–8]. Osteoprotegerin (OPG), as one member of the superfamily of tumor necrosis factor receptors, is the pivotal molecules in the ossific process and has been proved to be involved in calcification [9]. It has reported that the changes of OPG, receptor activator of nuclear factor-kB (RANK), and RANK ligand (RANKL) gene expression were observed in natural stenosis valves and biological valves [10, 11]. Meanwhile, OPG can inhibit RANK and its ligand RANKL, and promote bone demineralization and vascular calcification, indicating that OPG/RANK/RANKL pathway has potential involvement during arterial and valve calcification [10]. Nevertheless, it still has limited evidence that the interference of OPG/RANK/RANKL triad is existing in AS patients, and whether these mediators may actively facilitate valve calcification remains uncertain. In the present study, we aimed to investigate whether OPG/RANK/RANKL expression is modified in aortic valve tissue of AS patients with or without valve calcification.

## 2. Materials and Methods

### 2.1. Patients and Aortic Valve Tissue

Aortic valve samples were collected from 38 patients with AS (24 males and 14 females; aged 49-76 years, with an average of 65.79 ± 6.61 years) undergoing valve replacement in our hospital from June 2018 to December 2020. The diagnosis of aortic valve stenosis was based on the history of present disease, physical examination, chest X-ray, and color Doppler echocardiography. Patients were excluded if they had rheumatic diseases, moderate and severe aortic regurgitation, severe liver and kidney diseases (eGFR <60 mL/min/1.73 m^2^), autoimmune diseases, tumors and metastases, and endocrine and metabolic diseases. The study protocol was approved by the Ethics Committee of Tianjin Chest Hospital (No. 2021KY-010-01), and all patients signed informed consent. The tissue samples were excised from aortic valve leaflets, then washed with cold saline to remove blood, frozen in liquid nitrogen, and stored at -80°C. Partial frozen tissues fixed by formalin and embedded paraffin were cut into 5-*μ*m-thick slices for the following experiments.

### 2.2. Hematoxylin-Eosin (HE) Staining and Alizarin Red-S Staining

The tissue sections were defatted with xylene and hydrated through a graded series containing 100%, 85% and 70% ethanol, and washed twice by distilled water. For HE staining, briefly, the sections were stained by hematoxylin solution (Zhuhai Beso Biotechnology Co. Ltd., Zhuhai, China) for 3 mins, and counterstained by eosin solution (Zhuhai Beso Biotechnology Co. Ltd., Zhuhai, China) for 10 mins, finally dehydrated with gradient alcohol and sealed with xylene transparent. Meanwhile, the tissue sections were dyed with 2% alizarin red-S solution (PH 4.2; Shanghai Yuanye Biotechnology Co., Ltd., Shanghai, China) for 5 mins and then were carefully rinsed with double-distilled water and allowed to dry. A light microscope (DM2500, Leica, Germany) was used to observe the tissue sections and photographed.

### 2.3. Immunohistochemistry

Paraffin sections were dewaxed, washed with anhydrous alcohol for 3 times, and washed with phosphate-buffered saline (PBS, pH 7.5-7.7) for 3 times, treated with antigen repair buffer-EDTA (pH 9.0) at 100°C for 20 mins, and washed with PBS for 4 times. The sections were incubated in 0.3% endogenous peroxidase blocking solution for 5 mins and washed with PBS for 3 times. Following, the sections were incubated with the primary antibodies for 15 mins at room temperature and washed with PBS for 3 times. The primary antibodies were rabbit polyclonal antibodies against human RANKL and against human OPG or mouse monoclonal antibody against CD 68 (Beijing Biosynthesis Biotechnology Co., Ltd., Beijing, China; dilution 1 : 1000). After washing, the sections were incubated with a biotin-labeled secondary antibody for 8 mins. As chromogen, 3,3'-diaminobenzidine (DAB) was used for 5 mins. Cell nuclei were counterstained with Meyer's hematoxylin at room temperature for 5 mins. For quantification of immunostaining, the sections were examined and photographed in high-power fields at an original magnification of 100 (objective). For semiquantitative analysis of the pathological sections, 100-fold field images were taken by Leica microscope. Immunohistochemical images (×100) were taken from 10 different random fields of each sample. The results of immunohistochemistry were judged according to the intensity of staining: colorless was negative; light yellow was weak positive; brown-yellow was positive; and brown was strong positive (negative and weak positive results were statistically analyzed as negative).

### 2.4. Mass Spectrometry Methylation Assays

Primer design for methylation assays was performed using Agena Bioscience EpiDesigner software: 5′-AGGAAGAGAGAGGTATTTAAGGGTATTTTTGGTGG, 3′-CAGTAATACGACTCACTATAGGGAGAAGGCTCCTATAATCCCAACATTTTAAAAAACC. DNA was isolated from aortic valve tissue using plant DNA extraction kit (Bioteke, Beijing), and genomic DNA was treated with sodium bisulfite (NaHSO_3_) using the EZ DNA methylation kit (ZymoResearch, CA, USA) following the protocol supplied by the manufacturer. PCR reactions amplifying bisulfite-treated DNA are performed on an ABI MP-300V PCR system (Applied Biosystems, CA, USA) using Retroscript RT-PCR kit (Ambion, Inc., TX, USA) according to the manufacturer's instruction. The forward (0.2 *μ*L) and the reverse primers were (0.2 *μ*L) used in 200 nM Trisbase, 6.4 *μ*L ddH_2_O, 1 *μ*L 1 × 10 × PCR buffer, 1 *μ*L dNTPs, 5 U/*μ*L PCR enzyme, 0.2 *μ*L 0.4-0.6 unit/reaction, and 1 *μ*L DNA template in a 10 *μ*L vol. The reaction was denatured for 4 mins at 90°C and then thermocycled for 20 s at 94°C, 20 s at 56°C, and 30 s at 72°C 4 mins. After PCR thermal cycling, unincorporated dinucleotide triphosphates were removed by inducing shrimp alkaline phosphatase (SAP) treatment. The total volume for the SAP purification reaction was 7 *μ*L, including 3.21 *μ*L RNase-free ddH_2_O, 0.89 *μ*L 5× T7 polymerase buffer, 0.22 *μ*L T cleavage transcription mix, 0.22 *μ*L DTT, 0.40 *μ*L T7 RNA and DNA polymerase, 0.06 *μ*L RNase A (0.09 mg/mL), and 2 *μ*L PCR/SAP mix. Reaction conditions were 37°C for 3 h and 85°C for 5 mins. The PCR products were purified using resin, were spotted onto a chip by using the MassARRAY nanodispenser, and were analyzed on the MassARRAY® Analyzer 4 (Agena Bioscience, Inc., CA, USA).

### 2.5. Real-Time Quantitative PCR

RNA was extracted from human aortic valve tissue by TRIzol reagent (Ambion Inc., TX, USA). cDNA was prepared by reverse transcription with the RevertAid first-strand cDNA synthesis kit (Thermo Fisher Scientific, Waltham, MA, USA). Then, qRT-PCR was performed to detect the expressions of OPG and RANKL using the TB Green Premix Ex Taq (Tli RNaseH Plus, TaKaRa, Japan) on a 7500 real-time PCR system (Applied Biosystems, CA, USA). The qRT-PCR reaction mixture contains 7.6 *μ*L H_2_O, 10 *μ*L 2× SYBR Green Mix, 0.4 *μ*L ROX, 0.5 *μ*L forward primer (5 *μ*mol/L), 0.5 *μ*L reverse primer (5 *μ*mol/L), and 1 *μ*L cDNA in a 20 *μ*L vol. The reactive conditions were as follows: predenaturation, 95°C, 30 mins; denaturation, 96°C 5 mins; and annealing, 58°C, 34 mins, 40 cycles. The final relative expression of OPG and RANKL was calculated using the 2^*ΔΔ*Ct^ method and normalized to GAPDH. The primers were purchased from Invitrogen (Thermo Fisher Scientific, Inc., Shanghai, China). and shown as follows: OPG-F, 5′-GAGTCCGATCCAGCCAAGA-3′; OPG-R, 5′-GTACGGCGGAAACTCACAG-3′; RANKL-F, 5′-TCGCTGGGAAACAACACTG-3′; RANKL-R, 5′-GGGAAGGGAAAGGTAGATGC-3′; GAPDH-F, 5′-GGAGCCAAAAGGGTCATC-3′, GAPDH-R, 5′-CCAGTGAGTTTCCCGTTC-3′.

### 2.6. Enzyme-Linked Immunosorbent Assay (ELISA)

The thawed specimens were placed at room temperature for at least 30 mins and then homogenized with lysate. The corresponding ELISA kits (Elabscience Biotechnology Co., Ltd., Wuhan, China) was used to test the concentration of the OPG and RANKL following the instructions of manufacturer. The absorbance OD value was monitored at wavelength range of 450 nm by a microplate reader.

### 2.7. Statistical Analysis

SPSS22.0 software package was used for statistical analysis. The measurement data in accordance with normal distribution were expressed as mean ± standard deviation. *T*-test was used for comparison between groups, and *χ*^2^ test was used for counting data. *P* < 0.05 was considered statistically significant.

## 3. Results

### 3.1. Baseline Characteristics of Patients

After HE staining and alizarin red-S staining, the patients were divided into noncalcified group (*n* = 21) and calcified group (*n* = 17). HE staining showed that in the noncalcified group, the valve tissue structure was clearly layered, accompanied by inflammatory cell infiltration, but no calcification was observed; in the calcified group, the valve structures were destroyed, and many calcifications were observed (Figures 1(a) and 1(b)). Alizarin red-S staining was negative in the noncalcified group, while alizarin red-S staining was positive in calcified group (Figures 1(c) and 1(d)). There was no significant difference in terms of the clinical and biochemical parameters between the two groups (all *P* > 0.05, Table 1).

### 3.2. Results of Methylation and RT-PCR Assays

According to bioinformatics analysis, one CpG-rich region (19 CpG loci) was found in OPG gene, ranging from 187 bp to 567 bp, and two CpG-rich regions were found in RANKL gene: one upstream region (26 CpG loci), ranging from 416 bp to 875 bp, and one downstream (12 CpG sites), ranging from 502 bp to 736 bp (Figures 2(a) and 2(b)). Subsequently, CpG-rich regions of OPG and the downstream of RANKL were analyzed by mass spectrometry (Figure 2(c)). The results showed that there were significantly differences in the average methylation rate of OPG gene between noncalcified group and calcified group (14.59 ± 10.94% vs 7.42 ± 7.45%, *P* = 0.027). The overall methylation degree of RANKL gene was generally low, with an average methylation rate of 0.93%-9.00%, and was 6.88 ± 1.65% and 5.53 ± 1.87% in noncalcified group and calcified group, respectively, with significant differences (*P* = 0.025, Figures 3(a) and 3(d)).

RT-PCR analysis showed that the mRNA expression of OPG was significantly different between noncalcified group (5.4014 ± 4.7057) and calcified group (10.4488 ± 6.1165, *P* = 0.007, Figure 3(b)), and it was negatively correlated with the methylation rate of OPG gene determined by mass spectrometry (*R* = −0.359, *P* = 0.027, Figure 3(c)). The mRNA expression of RANKL was significantly different between noncalcified group (29.9071 ± 111.9302) and calcified group (116.5312 ± 133.8012, *P* = 0.036, Figure 3(e)), and it was also negatively correlated with the methylation rate of RANKL gene (*R* = −0.407, *P* = 0.011, Figure 3(f)).

### 3.3. Expression of OPG and RANKL in Aortic Valve Tissue

According to the immunohistochemical staining, OPG and RANKL were positively expressed in calcified aortic valves, while OPG and RANKL were not expressed in noncalcified aortic valves (Figures 4(a) and 4(b)). ELISA showed that the protein expression level of OPG (1.6697 ± 0.4839 ng/mL vs 2.1193 ± 0.4068 ng/mL, *P* = 0.004, Figure 4(c)) was obvious higher in noncalcified group compared with that in calcified group, while the protein expression level of soluble RANKL (sRANKL) was significant lower in noncalcified group compared with that in calcified group (0.0978 ± 0.0225 pg/mL vs 0.1159 ± 0.0303 pg/mL, *P* = 0.042, Figure 4(d)).

### 3.4. Expression of OPG and RANKL and Macrophage Infiltration

The macrophage infiltration and the expression of OPG and sRANKL in valve tissue were evaluated by immunohistochemical staining of CD68. Immunohistochemical staining showed that CD68-positive macrophages were preferentially associated with focal calcification, but were evenly distributed throughout the valve layers (Figure 5(a)). Furthermore, the ELISA results showed that the sRANKL level of CD68+ macrophages group (0.1243 ± 0.0321 pg/mL) was significantly different from that of CD68- group (0.0984 ± 0.0218 pg/mL, *P* = 0.007, Figure 5(b)). There was no significant difference in OPG level between CD68+ macrophages group (1.9411 ± 0.4554 ng/mL) and CD68- group (1.8422 ± 0.5218 ng/mL, *P* = 0.587, Figure 5(b)).

## 4. Discussion

The aortic valve leaflet is divided into three layers, and each layer is composed of valvular interstitial cells (VICs), extracellular matrix, and valve endothelial cells, without vascular tissue. Under normal physiological conditions, VICs is static, which is transformed into an activated phenotype after stimulated by lipid deposition, inflammatory response, oxidative stress, and other stimulation [12]. The expressions of *α*-smooth muscle action (*α*-SMA) and related signaling pathways are upregulated as a response, and pathological findings showed thickening of valve fibers. If the stimulation continues, VICs will continue to differentiate into osteogenic phenotypes and activate BMP-2, Runx2, and other important signal molecules closely related to osteoblasts [13], producing a series of calcification-related proteins, such as alkaline phosphatase, osteopontin, and osteocalcin, and eventually calcification [14], and the OPG/RANKL/RANK pathway is involved in this process. In this study, the calcified group and the noncalcified group were divided according to HE and alizarin red-S staining. The OPG/RANKL gene methylation, RT-PCR, immunohistochemistry, and ELISA were performed on the valve tissues of AS patients to preliminarily explore the influence of this signaling pathway on valve calcification.

RANKL can be generated by the osteoblast and T lymphocyte secretion. RANKL is the important regulatory factor for physiological bone formation and lymphocyte differentiation, it can promote cell proliferation, activate matrix metalloproteinases (MMP)-1 and MMP-2, and promote the transformation of stromal cells into osteoblast-like cells [15]. In addition, RANKL can also bind to RANK on the surface of osteoclasts and induce a series of reactions leading to bone tissue absorption and extracellular matrix degradation, which can destroy bone tissue in the presence of osteoblasts [16], indicating that RANKL is involved in various mechanisms of valve calcification. OPG regulates the differentiation and maturation of osteoclasts by competitively binding RANK with RANKL and participates in the formation and regulation of valve calcification in CAVD patients [17]. However, previous studies have shown inconsistent results on the expression of OPG in calcified valves [18, 19]. Therefore, the expression of OPG and RANKL in valve tissues was detected in this study, and it was found that the mRNA expression of OPG and RANKL, as well as the protein expression detected by immunohistochemistry or ELISA, was significantly increased in calcified valve tissues compared with noncalcified valve tissues.

The infiltrating inflammatory cells cannot be found in normal heart valve tissue, but be found in calcified valve tissue in the early stage, and these cells can release a variety of cytokines and growth factors by activating NOTCH, BMPs, Wnt, and NF-*κ*B and other signal transduction pathways to promote the occurrence of cardiac valve calcification [20]. Macrophages are the largest inflammatory cell group in calcified aortic valve disease [21]. RANKL is closely related to macrophages, which can be expressed by macrophages, mediates the migration of macrophages, and jointly regulates the differentiation and maturation of osteoclasts with OPG and rank on the premise of osteoblasts [16]. Therefore, in this study, CD68 staining of macrophages was also performed, and it was found that sRANKL value in the positive group was significantly higher than that in the negative group. However, no significant difference was found in OPG value between the two groups, indicating that there may be other reasons for the increase of OPG in valve tissues. DNA methylation is common in cardiovascular diseases, and the relationship between aortic valve calcification and methylation has been confirmed in recent studies [22, 23]. We speculate whether the reason for increased OPG expression is related to the degree of gene methylation. The degree of gene expression is closely related to the methylation status of DNA. The highly expressed genes tend to be hypomethylation, while the silenced genes tend to be hypermethylation. In this study, we observed that the methylation rate of OPG gene was significantly reduced in calcified group, and was negatively correlated with mRNA expression, thus confirming that the upregulation of OPG expression was related to gene methylation modification. The same changes also appeared in the detection of RANKL, but the methylation degree of RANKL gene was generally reduced. Whether it was the primary change or the secondary result remains to be further confirmed.

Several limitations of our work need recognition. Due to the small amounts of aortic valve samples from valve replacement, we could determine OPG expression and RANKL expression in aortic valve tissue only by using mRNA determinations and immunohistochemistry. Postoperative OPG and RANKL were not measured in all patients undergoing valve replacement. Thus, the OPG, RANKL variants, CD68 levels, and clinical parameters of patients were not compared in the result. Nevertheless, additional work will be required to confirm whether the degree of methylation of OPG and RANKL genes takes part in the regulation of valve calcification *in vivo.*

In conclusion, OPG and RANKL genes were hypomethylation in calcified valves, accompanied by the increase of corresponding mRNA and protein expression, suggesting that the degree of methylation of OPG and RANKL genes may play an important role in regulating valve calcification in AS patients.

## Figures and Tables

**Figure 1:** HE staining and alizarin red-S staining (magnification 100×). (a) HE staining in noncalcified group. (b) HE staining in calcified group. (c) Alizarin red-S staining in noncalcified group. (d) Alizarin red-S staining in calcified group.

**Figure 2:** (a) CpG-rich region in OPG gene. (b) CpG-rich region RANKL gene. (c) The methylation rate of OPG and RANKL genes determined by mass spectrometry.

**Figure 3:** Results of mass spectrometry methylation detection and RT-PCR of two groups. (a and d) Comparison of gene methylation rate between noncalcified group and calcified group. (b and e) Comparison of mRNA between the two groups. (c and f) Correlation between methylation rate and mRNA.^∗^*P* < 0.05, ^∗∗^*P* < 0.01.

**Figure 4:** Immunohistochemical staining and ELISA. (a) OPG immunohistochemical staining showed no positive staining in the noncalcified group and positive staining in the calcified group. (b) RANKL immunohistochemical staining showed no positive staining in the noncalcified group and positive staining in the calcified group. (c–d) ELISA showed significant differences in OPG and sRANKL levels between the two groups. Immunohistochemical staining, magnification 100×; ^∗^*P* < 0.05, ^∗∗^*P* < 0.01.

**Figure 5:** (a) CD68 immunohistochemical staining, negative and positive. (b) ELISA results showed that SRANKL level of CD68+ group was significantly different from that of CD68- group, but OPG level was not significantly different. Immunohistochemical staining, magnification 100×; ^∗^*P* < 0.05.

**Table 1:** Comparison of clinical and biochemical parameters in calcified group and noncalcified group.

Parameter	Noncalcified group (*n* = 21)	Calcified group (*n* = 17)	*P* value
Gender [*n*, (%)]			0.859
Male	13 (61.90%)	11 (64.71%)	
Female	8 (38.10%)	6 (35.29%)	
Age (year)	64.57 ± 7.35	67.29 ± 5.41	0.211
BMI (kg/m^2^)	25.14 ± 1.83	25.16 ± 1.41	0.974
Smoking [*n*, (%)]	9/42.86	7/41.18	0.917
CHD [*n*, (%)]	2/9.52	3/17.65	0.640
Hypertension [*n*, (%)]	10/47.62	9/52.94	0.744
Diabetes [*n*, (%)]	3/14.29	1/5.88	0.613
MVD [*n*, (%)]	2/9.52	1/5.88	1.000
LVEDD (mm)	57.76 ± 9.07	55.35 ± 7.64	0.389
Ejection fraction (%)	51.52 ± 12.57	56.94 ± 7.93	0.115
Aortic blood-flow velocity (m/s)	4.21 ± 0.85	4.66 ± 1.19	0.181
Mitral pressure gradient (mmHg)	46.33 ± 16.66	55.12 ± 26.02	0.239
Creatinine (mg/dL)	1.02 ± 0.32	0.98 ± 0.33	0.705
UA (*μ*mol/L)	299.14 ± 75.93	328.35 ± 139.93	0.447
LDL-C (mmol/L)	2.73 ± 0.67	3.03 ± 0.84	0.232
CRP (mg/L)	2.13 ± 2.10	2.50 ± 2.09	0.592
Medication therapy [*n*, (%)]			
ACEI	8 (38.10%)	7 (41.18%)	0.847
Antihypertensive drugs	5 (23.81%)	5 (29.41%)	0.727
Statins	6 (28.57%)	10 (58.82%)	0.060
Diabetes treatment	3 (14.29%)	1 (5.88%)	0.613

CHD: coronary heart disease; mitral valve disease; LVEDD: left ventricular end-diastolic diameter; UA: uric acid; LDL-C: low-density lipoprotein cholesterol; CRP: C-reaction protein; ACEI: angiotensin converting enzyme inhibitor.

## Data Availability

The data used to support the findings of this study are available from the corresponding author upon request.
